The article "The Psychological Recovery of Patients in the Context of Virtual Reality Application by a Complementary Medicine Scheme Based on Visual Art" was published in 2022. Journal: Evid Based Complement Alternat Med.

# The Psychological Recovery of Patients in the Context of Virtual Reality Application by a Complementary Medicine Scheme Based on Visual Art

**DOI:** 10.1155/2022/7358597

**Published:** 2022-09-19

**Authors:** Bolin Li, Meilin Shen

**Affiliations:** ^1^Shanghai University, Shanghai Academy of Fine Arts, Shanghai, China; ^2^Department of Publishing and Dissemination, Shanghai Publishing and Printing College, Shanghai, China; ^3^Department of Film and Television Art, Shanghai Publishing and Printing College, Shanghai, China

## Abstract

Expressive art therapy, which originated from art therapy, uses visual art as a carrier and plays a complementary role in clinical medicine and psychological medicine in the healing process of mentally ill patients. With the rapid development of science and technology, expressive art therapy has also entered the field of technology-oriented virtual reality. This study aims to summarize the clinical psychology research of expressive art therapy based on virtual reality, to review the current state of the field, in order to provide detailed scientific research evidence summary for relevant content and complete knowledge reserve.

## 1. Introduction

As one of the complementary treatments, expressive art therapy with visual art as a carrier originated from art therapy and first appeared in 1942 [1]. American psychiatrist Margaret Naumburg proposed the concept of art therapy and promoted the art therapy model establishment. In the 1950s, psychologists encouraged patients to use various artistic media to express their inner fears, depression, and contradictions during psychotherapy. Since then, expressive art therapy has become basic psychotherapy [2]. In the 1970s, expressive art therapy had a further development, and researchers found that it could activate patients' self-awareness and communication, enhance creativity, adjust their emotional state, help release emotions, and help achieve physical and mental healing. After participating in experiential therapy groups, many people suggested that the experience of therapy did have a positive impact on their mental health and social relationships. Because of these characteristics, expressive art therapy is now used in various fields, such as schools, hospitals, prisons, interventions, and rehabilitation training for special populations [1]. As a creative expression for therapy, expressive art therapy originates from the blending of art and psychotherapy. In a broad sense, it includes a variety of artistic means, such as painting, drama, and music., while in a narrow sense, it refers to painting-based visual art therapy, including sculpture, photography, and digital art [3, 4]. In this review, we focus on expressive art therapy in the form of visual arts.

## 2. Psychological Principles of Expressive Art Therapy

### 2.1. Principles of Psychoanalysis

The practice of art therapy emerged with the development of psychoanalytic theory. It combined free association, which is one of the main treatments of Freudian psychoanalysis, and the diagnosis and analysis of painting based on psychoanalytic theory [5]. It became an important theoretical basis for imagery connectivity in art treatment. Under the guidance of the theory of unconscious repression and the theory of collective unconscious imagery, Margaret Naumburg proposed art psychotherapy [6]. She encouraged the use of spontaneous artistic expression of consciousness as a medium of self-therapy to directly express dreams, illusions, and other inner experiences in the form of images rather than verbal language to solve the transference relationship in therapy and to transfer the patient's dependence on the therapist to artwork attention. Edith Kramer proposed art behavioral therapy based on Freud's psychoanalytic theory, emphasizing the use of art as a tool to purify emotions to help patients convert primitive impulses and illusions into artwork. At the same time, she paid more attention to improve the emotional and behavioral problems of children with special needs with the aid of artistic means and believed that through the specific presentation method of art in the creative process, it can help individuals find and sublime their inner real feelings and integrate reality and illusion and consciousness and unconsciousness, so as to achieve the effect of treatment [5].

### 2.2. Principles of Cognitive Development

With the development of cognitive behavioral therapy, cognitive behavioral art therapy with psychoeducation as the value orientation emerged, some scholars began to implement this cognitive behavioral therapy for patients with anxiety and panic disorders and proposed that psychological imagery can enhance patients' self-control, and emotional and behavioral problems can be improved in cognitive processes [7]. On the basis of child developmental psychology, Ron Field proposed that artistic expression has a positive effect on the emotional development of children with special needs and suggested that therapists design corresponding courses as needed from the perspective of children, so as to promote the development of their emotional functions, and proposed developmental extension from individual therapy to holistic rehabilitation education [5, 7].

### 2.3. Gestalt Psychology

Kurt Koffka proposed Gestalt theory and explained that human behavior is a kind of “field,” and it is divided into two major systems: one is the environment and the other is the self, and the two are inseparable. Gestalt psychology emphasizes that organisms perceive entire patterns or configurations, not merely individual components [8]. Gestalt principles, such as proximity, similarity, figure-ground, continuity, closure, and connection, describe how humans perceive visuals in connection with different objects and environments [9]. On the basis of Gestalt theory, Janie Rhyne proposed “Gestalt painting therapy,” which requires patients to perform a series of emotional experiences as complete Gestalt, such as abstract drawings on emotional experiences such as joy, fear, and anger [10], and each painting is not only a part of the whole but also a single Gestalt unit, and then by encouraging patients to illustrate, associate, and compare the similarities and differences of paintings, we find the crux of the painting and promote patient cognitive ability by review and discussion.

## 3. Advantages of Expressive Art Therapy

Expressive art therapy is a method that uses various media to help participants heal mental disorders, resolve conflicts, expand self-awareness, and thus achieve psychological healing [11]. In this safe, nonverbal healing environment, people's protective alertness is weakened, and participants' emotions can be soothed, resolved, and vented so that they can face themselves and others better and naturally express their inner feelings [12]. Therefore, expressive art therapy has the following advantages [13].

### 3.1. Nonverbal Communication

Expressive art therapy is not stressful for the participants, offers no restrictions on the participants' cognition, age, language, and art capabilities, enables self-creative expression in all possible ways, and has unique advantages for those unable to communicate or not good at talking [14].

### 3.2. Provide a Safe and Private Creative Healing Environment

This atmosphere helps reduce the psychological defense of the experiencer so that they can present the authentic self, while at the same time, it helps them present their inner thoughts and ideas through artistic expression on the artwork, which helps them recognize emotions and ideas, thereby promoting self-integration [15, 16].

### 3.3. The Function of Space-Time Integration

Through artistic expression, inner thoughts and emotions can be associated with different events at different times and places, and even contradictory emotions can be presented in the same work [17].

### 3.4. Easy and Effective Implementation

None of the materials and operating conditions required in the healing process are highly demanding, which can be carried out in all daily life situations, and they are intriguing and easy to operate [18].

## 4. Visual Art: An Important Carrier for Expressive Art Therapy

As the most important part of expressive art therapy, visual art focuses on the integration of thoughts and emotions, and the healing process is the expansion of consciousness. Humans can receive and feel external information through vision, smell, hearing, taste, and touch [19]. About 85% of external information is obtained through the eyes, that is, vision. Vision, as a dependent system, can only exhibit its healing properties when it has gained enough freedom. More and more exhibitions curated by museums now involve immersive experiences led by visual design. For example, the “Healing Art” theme exhibition held by Shanghai Liu Haisu Art Museum guides people to self-healing by various visual designs such as installation art, painting, and color so that art and design can soothe their emotions [20]. Based on the healing function of visual art and its gentle natural attributes, visual art can be applied in some public welfare projects, such as photography, handicraft, video, painting, design, and other forms to provide services and help for mentally handicapped persons [21].

In visual art therapy, color and graphics are used as research priorities in treatment programs, especially in the treatment of children. The psychological effect of color begins with a vision and encompasses psychological processes such as perception, emotion, memory, and thought. Different colors can have different effects on people's emotions, which are linked to people's life experiences and memories, and are able to produce color associations, thus causing changes in mood. Usually, red represents enthusiasm and festivity, and yellow represents brightness and lightness [22]. Dark colors, such as black and gray, give people a heavy and sad feeling. Studies have shown that blue can inhibit excitement, red can make people active in mental activities, and green can relieve tension. Therefore, color can enable patients to express and vent their emotions, meet their psychological needs, and intervene in patients' emotions [23]. Graphics is another important point in visual art treatment. Because visual activities are active and highly selective, participants can directly identify objects when perceiving graphics, especially flat graphics, and the rich combination of graphics can stimulate imagination [24]. Presenting an individual's inner feelings through the multiple combinations of graphics, as well as the expressivity of colors, helps regulate stress and soothe emotions.

Artists reproduce trauma through artistic works to achieve self-reflection and self-confidence and achieve self-healing of the body and mind. American artist Louise Bourgeois achieved self-healing through self-confession art. Her works were presented to the audience in the form of autobiographical stories, which contain the artist's spiritual trauma. In 1974, she created a composite sculpture “the Destruction of the Father” (Figure 1). In the dark, small, den-like space, there were many orange balls of latex on the ceiling and floor (Bourgeois's father had mocked her femininity with oranges), surrounding a rectangular dining table with various shapes destroyed by violence. This was her encounter with shadows in her personality through her sculpture creation. She subconsciously exposed the scenes that reproduced and exaggerated the painful memories of her childhood and expressed her resentment against her father in this way. The creative method is a self-healing of childhood pain. Louise Bourgeois also created the huge sculpture “Maman” series (Figure 2), and she believed that spiders have characteristics of mothers, who work in repairing blankets and textiles to make money and raise their children, just as spiders spin webs to protect baby spiders. She deliberately enlarged the size of the spider to a shocking level, not only for emotional satisfaction and transfer but also for showing the strength of women and encouraging herself to become stronger and fight for and defend her own rights. Japanese artist Yayoi Kusama is the first artist to make a mirror house. She persistently used the dot pattern to extend the space through mirror reflection, giving people a feeling of infinite proliferation, like entering a fantasy world (Figure 3). The dots are a way for Yayoi Kusama to express her mind in her artworks. Mirrors, as a tool for infinite repetition and reproduction of dots, are an indispensable element in her spiritual self-healing process.

## 5. Making Art Therapy Virtual: Integrating Virtual Reality into Art Therapy

Virtual reality is a computer-advancedhuman-machine interface with immersion, interactivity, and conception as the basic characteristics [3, 25]. It integrated the use of computer graphics, simulation technology, multimedia technology, artificial intelligence technology, computer network technology, parallel processing technology, and multisensor technology to simulate the functions of human sense organs such as vision, hearing, and touch so that people can immerse in the computer-generated virtual circle, interact with it in real time through natural ways such as language and gestures, and create an individualized and multidimensional information space [26]. Users can not only feel the immersive fidelity experienced in the objective physical world through the virtual reality system but also can break through space, time, and other objective constraints and feel the experience that cannot be experienced in the real world [27].

In recent years, some researchers have used VR as a psychotherapy tool and introduced it into expressive art therapy, especially for adolescents. Art therapy in VR can be thought of as a collage where images or selected parts of images are used, cut, and attached to new works that express different content, allowing people to re-express. Creation in VR combines elements of the painting (lines, patches, shapes, colors, and 2D), elements of the sculpture (3D), and novel elements supported by digital media [28]. This combination is similar to classical artwork but fundamentally different. The artwork itself is virtual and thus lacks concrete physicality and haptic feedback. The infinity, immersion, and dynamic environment of the virtual canvas can have a powerful impact on creators. Moreover, VR creation allows creators to observe the work from multiple angles, including from within the work itself [29]. VR creation requires a VR system (eg Oculus rift, HTC Vive) and a motion enclosure. Creators can move freely in the immersive 3D space, and the visual background of the environment can also be easily changed. Ohrius and Malchiodi studied the interaction and senses of digital media and argue that there is a clear difference between the sensory experience provided by digital technology and the traditional material approach, making digital media a viable alternative [30].

Instances of psychological recovery of patients in the context of virtual reality application by complementary medicine scheme based on visual art, Shamri Zeevi [25] used VR device, let participants wear a Head Mounted Display (HMD) and use Tilt Brush software by Google, also with two MOCAP, to creat artwork in the virtual space, the participants faced to a 3D space meanwhile the therapist faced to a 2D monitor. The therapist and the participants had no eye contact but only while speaking, and the purpose of the therapy was to reproduce and shape the psychological process of the patient through the process of creating works in the virtual world. Hacmun [3] presented a similar clinical method but was more focused on presence and immersivity.

Overall, VR technology may be particularly beneficial for adolescents who are refractory to traditional art treatments. VR can also be a therapeutic option for patients who are afraid of committing mistakes and are unable to try, as it allows experiential exploration without any impact on the physical or real world. For patients who do not consider themselves imaginative, VR art therapy can help them broaden their specific ideas and find ways to express themselves.

## Figures and Tables

**Figure 1:** Louise Bourgeois, the Destruction of the Father, 1974, Foto Lucie.

**Figure 2:** Louise Bourgeois, Maman Spider, 1999, Long Museum West Bund, Shanghai, 2018.

**Figure 3:** Yayoi Kusama, the Spirits of the Pumpkins Descended into the Heavens.

## Data Availability

There are no data used to support this study.
